The article "Diagnostic Value of Hcy Combined with Blood Pressure Variability Index in the Severity of Hypertension Complicated with CSVD and Its Correlation with Cognitive Function and CysC Expression" was retracted in 2023. Reasons: unreliable results or conclusions; lack of ethics approval or compliance; concerns about the data; concerns about the peer review.

# Diagnostic Value of Hcy Combined with Blood Pressure Variability Index in the Severity of Hypertension Complicated with CSVD and Its Correlation with Cognitive Function and CysC Expression

**DOI:** 10.1155/2022/9003537

**Published:** 2022-04-14

**Authors:** Qiaoling Liu, Xia Liu, Xuelian Zhang, Chen Zhou

**Affiliations:** ^1^Department of Geriatrics, The First People's Hospital of Lianyungang, Lianyungang, China; ^2^Xuzhou Medical University Affiliated the Hospital of Lianyungang, The First Affiliated the Hospital of Kangda College of Nangjing Medical University, Jiangsu 222000, China; ^3^Drug Clinical Experimental Center, The First Affiliated Hospital of Nanjing Medical University (Jiangsu Province Hospital), Nanjing, Jiangsu 210029, China

## Abstract

This paper explores the diagnostic value of Hcy combined with the blood pressure variability index in the severity of hypertension complicated with CSVD and its correlation with cognitive function and CysC expression. 200 patients with ischemic small cerebral vessels are selected as the research object. According to the MRI findings, they are divided into 48 cases of white matter lesions (WML), 44 cases of lacunar infarction (LI), 44 cases of enlarged perivascular spaces (EPVs), and 46 cases in the mixed group (referring to two or more types of ischemic cerebrovascular disease on imaging). Different cognitive domains of different types of ischemic cerebrovascular diseases are analyzed. The risk factors of cognitive decline in patients with ischemic cerebrovascular disease are analyzed by univariate analysis and multivariate logistic regression analysis. There is an ancestral correlation between serum Hcy and CSVD, which is an independent risk factor for CSVD.

## 1. Introduction

The global burden of ischemic stroke is almost four times that of hemorrhagic stroke. Current evidence suggests that 25–30% of ischemic stroke survivors develop immediate or vascular cognitive improvement (VCI) or vascular dementia (VAD). Poststroke dementia may include all types of cognitive impairment [1]. Prestroke cognitive impairment status is classified as prestroke dementia, which may lead to vascular changes and potential neurodegenerative processes. The risk factors of prestroke cognitive impairment and dementia are multifactorial, including old age, family history, genetic variation, low education level, systemic vascular disease, previous transient ischemic attack or recurrent stroke, and depression [2]. Until recently, cerebral small vessel disease (CSVD) proposed that cerebral small vessel disease is a common cerebrovascular disease, which refers to the disease based on intracranial vascular disease [3]. In various pathological and neural processes, it also refers to a syndrome with different clinical manifestations and the structural changes of blood vessels and brain parenchyma caused by neuroimaging features [4]. Small vessel disease accounts for 25% of all diseases, and the risk of ischemic stroke is twice that of general stroke. Cerebrovascular disease is the main cause of neurological loss, disability, and cognitive impairment. Cerebrovascular disease is closely related to age [5].

Therefore, with age, CSVD gradually leads to cognitive, mental, and physical dysfunction in many elderly people and increases the incidence of stroke. With the popularization and wide application of neuroimaging technology, a large number of small cerebrovascular diseases have been identified and found, which is of great significance for the prevention and treatment of small cerebrovascular diseases [6]. Cerebrovascular diseases have different meanings in different classification methods, and the pathological mechanism of microvessels is also different in different types of cerebrovascular diseases [7]. In addition, in order to clarify the cytomolecular mechanism of different types of cerebrovascular diseases, it is very important to understand the genetics behind the pathology of cerebrovascular diseases. Cognitive impairment is a neurological disease characterized by visuospatial executive ability and memory, which cannot be explained by other cerebrovascular diseases [8]. Mild cognitive impairment does not affect life and is difficult to judge clinically. Severe cognitive impairment can affect daily life and social activity. Previous studies have confirmed that lacunar infarction (LI) can increase the risk of dementia, especially the new lacunar infarction, which mainly damages the overall cognitive function and the psychomotor rate of patients, doubling the risk of dementia [9]. By analysing the risk factors related to different types of CSVD and the characteristics of cognitive impairment, this paper discusses the risk factors of cognitive decline in patients with ischemic cerebrovascular disease. This study aims to provide new ideas and methods for the clinical diagnosis and treatment of ischemic cerebrovascular disease and to provide a theoretical basis for the development of therapeutic drugs.

The rest of this paper is organized as follows: Section 2 discusses related work, followed by the proposed method designed in Section 3.  Section 4 shows the experimental results, and Section 5 concludes the paper with summary and future research directions.

## 2. Related Work

In recent years, many scholars at home and abroad have made a new understanding of cerebrovascular disease through in-depth research on cerebrovascular disease. At present, there is no ideal method for treating small vessel disease and cognitive decline at home and abroad. Therefore, it is important to further explore the risk factors of cognitive decline in patients with cerebral small vessel disease and to intervene actively to reduce the incidence rate [10]. Lacunar infarction and white matter lesions are described as recessive cerebrovascular diseases in people without a history of stroke, but they have important clinical consequences. It is associated with a 2–4-fold increase in the risk of clinically defined ischemic stroke, independent of vascular risk factors, and a 2–3-fold increase in the risk of dementia [11]. They may also directly destroy the functional network in the brain, leading to defects affecting cognition, gait, and other functions. Hcy is a nonessential amino acid sulfur produced by methionine metabolism, which is prone to self-oxidation and produce a variety of strong oxides. Wang et al. demonstrated that the Hcy level is closely related to ischemic cerebrovascular diseases, especially white matter lesions and lacunar infarction, and is regarded as an independent risk factor [12]. Data show that the high Hcy level is closely related to ischemic stroke. Some studies have confirmed that hyperhomocysteinemia is closely related to the occurrence and development of atherosclerosis and thromboembolic diseases. It is an independent risk factor of ischemic stroke [13]. When the body has functional metabolism disorder, Hcy accumulates in the body because of its inability to degrade, resulting in hyperhomocysteinemia. Hyperhomocysteinemia can promote vascular endothelial dysfunction through oxidative stress, increase blood coagulation, over activation of inflammatory response, atherosclerosis, and other processes, so as to promote the occurrence of ischemic cerebrovascular disease [14]. As an independent risk factor of ischemic cerebrovascular disease, the influencing factors of Hcy on WML may be greater than Li. The higher its level, the more serious the degree of WML. The results of this study found that the increase of the Hcy level is a risk factor for cognitive impairment in patients with ischemic cerebrovascular disease. After being included in logistic regression analysis, Hcy lost its predictive value [15].

WMH is the most common manifestation of CSVD on MRI, which is highly correlated with age and widely exists in patients with normal blood pressure [16]. Some scholars have suggested that the Hcy level may be an independent predictor of white matter lesions, which is positively correlated with the volume of white matter lesions in stroke patients. The smooth curve of this study shows that there is a significant difference in the effect of Hcy in patients with hypertension and nonhypertension. In the population with hypertension, the effect of Hcy on WMH is a persistent linear relationship [17]. It is speculated that the reason may be due to the joint action of Hcy and hypertension. In the nonhypertensive population, the influence of Hcy on WMH shows a “U” curve, and the influence before and after the turning point is quite different. Combined with the results of multivariate regression analysis, when Hcy ≥ 10 *μ*mol/L, Hcy increases by 1 *μ*mol/L, ARWMCs increased by 0.7 points. When Hcy < 10 *μ*mol/L, Hcy has no significant correlation with ARWMCs, that is, in nonhypertensive CSVD patients, the effect of high Hcy on brain white matter is significantly positively correlated and exists independently of hypertension [18]. Brain white matter is an important part of the central nervous system and a place where nerve fibers gather. Brain white matter lesions caused by demyelination can lead to motor, sensory, and cognitive impairment. Previous studies have suggested that the increase of plasma Hcy is an independent risk factor for cardiovascular and cerebrovascular diseases, which increases the risk of atherosclerotic vascular diseases by 2∼3 times, and Hcy > 14 *μ*mol/L, the risk of Alzheimer's disease increased by 1.8 times [19]. Hcy > 16 *μ*mol/L increased the risk of stroke by 87%; Hcy > 18 *μ*mol/L increased the prevalence of hypertension three times. Hypertension and age are the most important risk factors for white matter lesions. This study found that Hcy ≥10 in nonhypertensive patients *μ*mol/L increases the risk of leukoencephalopathy in patients, which is independent of age and hypertension. The effect of high Hcy on cerebral small vessel disease is greater than that of large vessel disease [20]. The possible mechanisms are as follows: (1) vascular endothelial toxicity; (2) dysfunction of vasomotor regulation and inhibition of cerebral small vessel dilatation; (3) promote the proliferation of small vascular smooth muscle cells, increase arterial stiffness, and even small cerebral vascular occlusion; (4) destroy the function of blood-brain barrier, increase the permeability, overflow plasma components, and damage small cerebral vessels; (5) the imbalance between the generation of free radicals and the antioxidant capacity of the body affects the redox signal pathway of blood vessels and nerve cells, resulting in neurological dysfunction; (6) make coagulation and lipid metabolism function abnormal, lead to lipid stripe disease and the formation of fibrous plaque, and accelerate the formation of atherosclerotic plaque; and (7) inhibit the activity of angiotensin-converting enzyme in endothelial cells, affect the physiological function of cerebrovascular and abnormal cerebral hemodynamics, and accelerate the process of cerebrovascular diseases. These mechanisms are independent of hypertension. Therefore, for nonhypertensive patients, when the plasma Hcy level reaches a certain level for a long time, it can theoretically lead to brain white matter injury [21].

Many studies have confirmed that WML, Li, and EPVs are related to cognitive decline, especially in executive function. Therefore, the impact of total CSVD and cognitive decline is positive. CSVD total load, as an indicator of the severity of cerebrovascular disease, has been widely used in clinical research [22]. Studies have confirmed that its severity is positively correlated with cognitive decline. Banerjee et al. conducted MRI analysis and cognitive evaluation analysis on 243 patients with mild cognitive impairment, cortical atrophy, and vascular dementia. Using multiple linear regression analysis, the results showed that the total load of CSVD is related to cognition, cortical atrophy, and intracerebral fiber injury. This study confirmed that the increase of CSVD total load is an independent risk factor for cognitive decline in patients with ischemic cerebrovascular disease, and the increase of CSVD total load is significantly negatively correlated with MOCA score, indicating that the heavier the degree of ischemic cerebrovascular disease, the more obvious the cognitive decline. Ischemic cerebral small vessel disease is not easy to detect and has a high incidence rate [23]. It can intervene in early stage of cognitive impairment by drugs, which can help patients to delay cognitive decline. As for the improvement of cognitive function, statins are selected to improve the blood lipid level, mainly because ischemic cerebrovascular disease occurs in the hypoperfusion of cerebral blood flow, microembolic embolism, and ischemic injury. The cholesterol in patients is high, and there is lipid hyaline or cellulose degeneration on the vascular wall of small blood vessels, which will lead to abnormal metabolism of brain tissue and damage to neurological function [24]. Therefore, statins are selected to improve the blood lipid level of patients in order to improve cognitive impairment. Statins can reduce the occurrence of vascular diseases and effectively prevent the decline of cognitive function. At the same time, atorvastatin is lipophilic and can inhibit the key enzyme hydroxymethylglutaric coenzyme A reductase in cholesterol synthase. The two are competitive, which limits the synthesis of cholesterol. In addition, atorvastatin protects endothelial function; has anti-inflammatory, antithrombotic, and antioxidant effects; and can protect neurological function through lipid-lowering effect, delay the progress of cognitive impairment, and prevent the occurrence of Alzheimer's disease to a certain extent. Ischemic cerebrovascular disease is characterized by concealed and diverse clinical manifestations, which not only cause stroke but also significantly affect the cognition, emotion, and daily living ability of patients. The incidence rate is on the rise [25]. In short, ischemic cerebrovascular disease is a common problem that affects the health of the elderly. Prevention of cerebrovascular diseases at the first and two levels is the key to reduce the incidence rate, recurrence rate, and disability rate of cerebrovascular diseases. Among the possible risk factors, age cannot be intervened but blood pressure, blood glucose, homocysteine, blood lipid, and other indicators can be intervened [26].

## 3. The Proposed Method

### 3.1. Research Object

This study is a cross-sectional study. 200 patients with ischemic cerebrovascular disease hospitalized in the Department of Neurology of our hospital from October 2019 to October 2020 are collected as the research object, and 50 normal people without abnormal outpatient imaging in the same period are collected as the control group. All subjects voluntarily participated in this study, accepted the questionnaire survey of cognitive score scale, improved the corresponding laboratory and imaging examination, and can provide complete research data.

### 3.2. Data Collection

The general data of patients with ischemic cerebral vascular disease and control group are collected, including gender, age, smoking history (1 cigarettes per day, 1 years and above), smoking history, drinking history (1 times a week, half a year or more as drinking), hypertension, diabetes, coronary heart disease, hyperlipidemia, carotid plaque, and past stroke history. Fasting white blood cells (WBC), neutrophils (NEU), lymphocytes (lym), platelets (PLT), mean platelet distribution volume (MPV), cholesterol (CHO), triglycerides (TG), high-density lipoprotein (HDL-C), low-density lipoprotein (LDL-C), uric acid (UA), apolipoprotein A (ApoA), apolipoprotein B (apoB), lipoprotein (LP), lipoprotein-associated phospholipase A2 (Lp-PLA2) and blood homocysteine (Hcy), and neutrophil lymphocyte ratio (NLR) and platelet lymphocyte ratio(PLR) are calculated.

### 3.3. Assessment of Cognitive Function

Cognitive impairment refers to the functional impairment of patients in higher cortical functions such as attention, memory, speech, thinking, and perception caused by organic diseases of the brain, such as stroke, tumor, and trauma. The Chinese version of Montreal Cognitive Assessment Scale (MoCA) is used in this study. The scale is revised by Nasreddine, clinical research center of Neurology, Charles Le Moyne hospital, Canada, based on clinical experience and referring to MMSE's cognitive item setting and scoring criteria. The score of Montreal Cognitive Assessment (MoCA) scale is evaluated by two neurophysicians with professional knowledge of neuropsychiatry. The total score <26 indicates cognitive impairment. The total score of those with education years ≤12 years is added by 1 point to correct the bias of education years. The lower the score, the heavier the cognitive decline. MOCA includes eight cognitive domains: visual space and executive function (5 points), memory (5 points), language (3 points), naming (3 points), attention (3 points), abstract thinking (2 points), calculation (3 points), and orientation (6 points). There are 11 inspections in total, with a total score of 30 points, which will be completed in about 10 minutes. There are 48 cases in the WML group, 44 cases in the Li group, 44 cases in the EPVs group, 46 cases in the mixed group, and 46 cases in the normal control group.

### 3.4. Statistical Methods

All statistical analysis is completed by SPSS 20.0 software. The measurement data conforming to the normal distribution are expressed in (*x* ± *s*). The comparison between multiple groups adopts one-way ANOVA, and the comparison between measurement data groups is subject to *t*-test. Analysis of counting data *χ*^2^ test, and the factors with statistical significance in univariate analysis are analyzed by multivariate logistic regression analysis. The difference is statistically significant (*P* < 0.05).

## 4. The Comparison of Experimental Results

### 4.1. Comparison of Clinical Data of Patients in Each Group

Compared with the control group, the proportion of hypertension and diabetes in patients with WML group, LI group, and EPVS group is higher. Age, TC, TG, LDL-C, Hcy, and D-two dimer levels increased significantly, and the level of LDL-C decreased (<0.05). Compared with a mild group, the proportion of male, hypertension and diabetes increased in severe group. Age, TC, TG, LDL-C, Hcy, and D-two dimer level increased significantly, and HDL-C level decreased (*P* < 0.05).  Table 1 presents the comparison of patient clinical data for each group.  Figure 1 shows the comparison of the clinical data of the patients in each group.

### 4.2. Comparison of MOCA Scores in Each Group

The total score of MOCA and the scores of cognitive domains in the mixed group are lower than those in WML group, Li group, and EPVs group. There is no significant difference in MOCA score and cognitive domain score among WML group, Li group, and EPVs group.  Table 2 presents the comparison of the MoCA scores in each group.

### 4.3. Comparison of Risk Factors between Cognitive Decline Group and Cognitive Normal Group

Univariate analysis showed that the total load of education, hypertension, carotid plaque, LDL-C, apoB, Hcy, and CSVD may be related to the decline of cognitive function in patients with ischemic cerebrovascular disease. The statistically significant variables in the univariate analysis results are included in the multivariate logistic regression analysis. The results showed that hypertension and the increase of CSVD total load are the risk factors for the decline of cognitive function in ischemic cerebrovascular disease.  Table 3 presents the comparison of risk factors between cognitive decline and cognitive normal groups.  Table 4 presents the multivariate analysis affecting cognitive decline in patients with CSVD.

### 4.4. Relationship Curve between Hcy and CSVD Brain White Matter

After adjusting age, gender, fasting blood glucose, glycerol three fat, total cholesterol and diabetes history, and the smooth curve of Hcy and ARWMCs fitted that Hcy and ARWMCs showed a U type relationship in nonhypertensive population, with a turning point of 10 *μ*mmol/L. In hypertensive population, Hcy and ARWMC showed an approximate linear relationship.  Figure 2 shows the relationship curve between Hcy and CSVD brain white matter.

## 5. Conclusion

This paper is a cross-sectional study. WML, Li, and EPVs are screened and evaluated by 1.5 T brain MRI. The subjects are scored with MOCA by professionals to evaluate their cognitive function. Foreign studies have found that Hcy may be related to the occurrence of cerebrovascular disease. Domestic studies have also found that Hcy is related to acute cerebral infarction, while there are few studies on the correlation of cerebrovascular disease. It is proposed that Hcy is related to cognitive impairment and innovative. However, this study involves the score of cognitive function scale, which may be subjective bias and interfere with the research results. At the same time, this study is a single-centre and small sample size study, and the conclusions still need to be further verified by larger sample and multicentre studies.

## Figures and Tables

**Figure 1:** Comparison of the clinical data of the patients in each group.

**Figure 2:** Relationship curve between Hcy and CSVD brain white matter.

**Table 1:** Comparison of patient clinical data for each group.

Index	WML group (*n* = 48)	LI group (*n* = 44)	EPVS group (*n* = 44)	Control group (*n* = 46)	*F*	*P*
Gender						
Female	21	20	18	19	0.250	0.969
Male	27	24	26	27		
Age	54.63 ± 7.12	62.03 ± 5.45	64.85 ± 5.25	59.32 ± 6.13		
Diabetes mellitus						
Yes	21	15	17	13	2.636	0.451
No	27	29	27	33		
TC (mmol/L)	4.69 ± 0.85	5.37 ± 1.03	6.14 ± 0.95	4.54 ± 0.71	12.562	0.004
TG (mmol/L)	1.95 ± 0.86	2.18 ± 1.03	2.51 ± 1.09	1.85 ± 0.92	4.268	0.041
HDL-C (mmol/L)	1.52 ± 0.40	1.38 ± 0.35	1.24 ± 0.29	1.69 ± 0.58	3.125	0.048
LDL-C (mmol/L)	2.42 ± 0.73	2.74 ± 0.75	3.35 ± 0.84	2.23 ± 0.58	3.351	0.043
Hcy (mmol/L)	10.76 ± 3.69	13.52 ± 2.41	16.15 ± 4.21	8.14 ± 2.14	15.201	0.000
D-dimer (mmol/L)	1.07 ± 0.13	1.83 ± 0.25	2.39 ± 0.42	0.43 ± 0.06	8.512	0.000

**Table 2:** Comparison of the MoCA scores in each group.

Index	WML group	LI group	EPVS group	Mixed group	*F*	*P*
MoCA score	21.3 ± 3.8	22.9 ± 4.6	23.5 ± 4.7	13.4 ± 5.8	26.541	0.000
Visual-space execution capability	2.9 ± 1.3	3.2 ± 1.5	3.2 ± 1.5	2.2 ± 1.4	14.521	0.000
Nominate	2.7 ± 0.6	2.8 ± 0.7	2.7 ± 1.5	2.3 ± 0.8	5.751	0.000
Memory	2.1 ± 1.8	2.6 ± 1.8	2.7 ± 1.5	1.0 ± 1.4	25.633	0.000
Count	2.5 ± 1.2	2.8 ± 0.8	2.7 ± 0.8	1.7 ± 1.2	8.110	0.000
Attention	1.6 ± 0.8	2.9 ± 0.8	2.8 ± 1.9	2.1 ± 0.9	7.658	0.000
Language	1.6 ± 0.8	1.9 ± 0.9	2.2 ± 1.0	1.3 ± 0.7	14.120	0.000
Abstract	1.2 ± 0.8	1.4 ± 0.9	1.5 ± 0.7	0.8 ± 0.7	13.326	0.000
Directive force	5.7 ± 0.8	5.6 ± 0.9	5.7 ± 0.9	5.8 ± 1.0	5.320	0.000

**Table 3:** Comparison of risk factors between cognitive decline and cognitive normal groups.

Index	Cognitive decline group	Noncognitive decline group	*t*	*P*
Age	68.12 ± 8.25	61.03 ± 4.98	8.325	0.014
NEU (×10^**9**^/L)	5.33 ± 2.28	5.46 ± 2.36	0.214	0.735
LYM (×10^**9**^/L)	1.52 ± 0.56	1.53 ± 0.54	0.196	0.974
MPV (fL)	10.65 ± 2.14	10.43 ± 1.58	1.412	0.098
NLR	4.35 ± 3.69	4.41 ± 3.02	0.226	0.932
PLR	180.32 ± 105.03	174.52 ± 111.84	0.126	0.714
TG (mmol/L)	1.50 ± 0.82	1.42 ± 0.85	0.295	0.595
CHO (mmol/L)	3.97 ± 0.93	4.26 ± 1.02	0.378	0.075
HDL-C (mmol/L)	1.15 ± 0.26	1.22 ± 0.40	4.216	0.201
LDL-C (mmol/L)	2.36 ± 0.83	2.76 ± 0.87	0.067	0.004
APOA (g/L)	1.38 ± 0.31	1.43 ± 0.32	0.416	0.652
APOB (g/L)	0.81 ± 0.24	0.92 ± 0.23	0.000	0.005
Hcy (mmol/L)	20.14 ± 7.94	17.08 ± 7.35	0.693	0.018

**Table 4:** Multivariate analysis affecting cognitive decline in patients with CSVD.

Index	*β*	SE	Wald	*P*	OR	95%CI
Age	1.526	0.103	8.345	0.013	1.725	1.025∼2.013
TG	1436	0.206	12.521	0.005	3.365	2.365∼7.820
LDL-C	1.521	0.562	29.365	0.001	3.521	2.541∼8.502
Hcy	0.869	0.320	24.521	0.001	2.698	1.684∼6.521

## Data Availability

The simulation experiment data used to support the findings of this study are available from the corresponding author upon request.
